The article "A Framework for Automatic Burn Image Segmentation and Burn Depth Diagnosis Using Deep Learning" was published in 2021. Journal: Comput Math Methods Med.

# A Framework for Automatic Burn Image Segmentation and Burn Depth Diagnosis Using Deep Learning

**DOI:** 10.1155/2021/5514224

**Published:** 2021-04-07

**Authors:** Hao Liu, Keqiang Yue, Siyi Cheng, Wenjun Li, Zhihui Fu

**Affiliations:** ^1^Key Laboratory of RF Circuits and Systems, Ministry of Education, Hangzhou Dianzi University, Zhejiang, China; ^2^The People's Hospital of Jianggan District, Hangzhou, Zhejiang, China

## Abstract

Burn is a common traumatic disease with high morbidity and mortality. The treatment of burns requires accurate and reliable diagnosis of burn wounds and burn depth, which can save lives in some cases. However, due to the complexity of burn wounds, the early diagnosis of burns lacks accuracy and difference. Therefore, we use deep learning technology to automate and standardize burn diagnosis to reduce human errors and improve burn diagnosis. First, the burn dataset with detailed burn area segmentation and burn depth labelling is created. Then, an end-to-end framework based on deep learning method for advanced burn area segmentation and burn depth diagnosis is proposed. The framework is firstly used to segment the burn area in the burn images. On this basis, the calculation of the percentage of the burn area in the total body surface area (TBSA) can be realized by extending the network output structure and the labels of the burn dataset. Then, the framework is used to segment multiple burn depth areas. Finally, the network achieves the best result with IOU of 0.8467 for the segmentation of burn and no burn area. And for multiple burn depth areas segmentation, the best average IOU is 0.5144.

## 1. Introduction

A burn is a common traumatic disease, usually caused by physical or chemical factors, such as heat, chemicals, electricity, or radiation. Small burns may cause damage to the skin and mucous membrane. Major burns may cause different degrees of functional, metabolic, and morphological changes in various systems of the body, resulting in severe pathological reactions, visceral damage, and other complications, with high mortality. Meanwhile, treatment process of burns is complex and takes a long time. Early treatment of burns has been proved to reduce the medical cost of patients [1]. With more and more attention paid to early burn treatment, early diagnosis of burn depth is more and more necessary. Accurate assessment of the burn area and depth to support reliable diagnosis is critical to the success of treatment and, in some cases, may save life of patients. In general, the depth of burns can be divided into superficial (first degree), superficial partial thickness (second degree), deep partial thickness (second degree), full thickness (third degree), and fourth degree [2]. The percentage of partial-thickness or full-thickness burns in the total body surface area (TBSA) is used to measure the burn size.

Usually, burn depth diagnosis is difficult to ordinary nurses or doctors but needs to be completed by clinical experts in burns. Doctors who are not burn experts may achieve less accuracy in assessing the depth of burns [3]. Clinical diagnosis by eye observation and physical examination is the most commonly used method to evaluate the depth of burns [4]. The visual assessment attempts to determine the depth of the burns and estimate the burn size in terms of TBSA. In order to achieve precise burn depth assessment, laser Doppler imaging [5], harmonic ultrasound imaging [6], optical coherence tomography [7], and high-resolution infrared thermography [8] have been developed and introduced into limited clinical diagnosis of burns. However, these devices are usually expensive and difficult to use and will not be widely adopted in clinic. A simple way to get burn images is through common cameras and smart phones. Then, the deep learning method may be used to diagnose and evaluate the depth of burn area. So far, the deep learning method has achieved excellent results in image classification and segmentation. Through deep learning technology, the burn image segmentation and burn depth classification can realize the automatic process of burn assessment, reduce the impact of human error, and improve the accuracy of visual assessment. Also, deep learning may reduce the cost of burn depth assessment and the time of diagnosis.

In this paper, in order to solve the problem of detecting the burn wound area and diagnosing burn depth from burn images obtained by using a camera or smartphone, an end-to-end framework for burn area segmentation and burn depth classification is proposed. The main contents of this paper are the establishment of the burn database, preprocessing and labelling of burn images, data augmentation of burns, and segmentation and classification networks of burn depth. The segmentation and classification models adopt fully convolutional networks and consist of an encoder and decoder. The encoder networks are used to extract the feature map of burn images, and the decoder networks are used to fuse and restore the feature map to input image size. Different backbone networks have been used to the encoder and decoder networks. Then, we use data augmentation and fusion loss function to train backbone networks. The networks are used for the segmentation and classification of burns. Finally, several metrics are used to evaluate the performance of burn image segmentation and depth classification. The results of the networks are visualized to analyze the performance on the test dataset.

The main contributions of this paper are as follows: (1) building a large labelled and segmented burn images dataset, (2) using novel data augmentation methods to improve the performance of the network, (3) using hybrid loss functions to train the networks, and (4) creating an end-to-end burn image segmentation and classification system, which has more clinical application.

## 2. Related Work

In the early study of burn depth, Serrano et al. [9] used the fuzzy-ARTMAP neural network to classify superficial dermal, deep dermal, and full-thickness burns. An average classification success rate of 88% was achieved. Wantanajittikul et al. [10] used *h*-transformation and texture analysis to extract feature vectors. Then, the support vector machine (SVM) was applied to identify the depth of burn and yielded the best results of 89.29% correct classification on the validation sets. Acha et al. [11] proposed a *k*-Nearest Neighbor (*k*-NN) classifier and obtained a success rate of 83.8% when classifying burns into three burn depths by using 74 images.

Recently, the convolutional neural network (CNN) has achieved great success in the task of general visual recognition and detection [12]. Therefore, more and more researchers try to apply CNN to burn images.

Badea et al. [13] proposed a convolutional neural network to identify burn areas from color image patches. And the network was proven to match the expected average precision of a trained burn surgeon. They split the burn area into 32 × 32 sized patches and trained the network to categorize each patch. They achieved overall precision of 75.91%. Despo et al. [14] proposed a fully convolutional network- (FCN-) [15] based network for automatic assessment and diagnosis of burn depth. Firstly, the image area was divided into the burn area and no burn area to verify the performance of the network in binary classification. By adding conditional random field (CRF) layer to based FCN and data augmentation, they achieved a pixel accuracy of 0.85 and intersection-over-union of 0.67. Then, the network was applied to multiburn segmentation. The multiburn network achieved pixel accuracy of 0.6 and mean intersection-over-union of 0.37. Finally, Despo et al. adopted the method of upsampled. And mean intersection-over-union was increased to 0.39, but the pixel accuracy was reduced to 0.57. Jiao et al. [16] designed a deep learning segmentation framework based on the mask regions with the convolutional neural network (mask R-CNN). They labelled 1150 images with the format of the Common Objects in Context (COCO) dataset and trained the model on 1000 images. And Jiao et al. compared different backbone networks in the framework. Finally, they used the Dice coefficient value to evaluate the model and achieved the average Dice coefficient of 84.51.

## 3. Methods

The framework of deep learning burn diagnosis is shown in Figure 1. It contains the following parts: the dataset of burn images, data augmentation, end-to-end burn depth segmentation networks, and result visualization. First, the burn images dataset is created. And we preprocess the burn images (crop and resize) and use data augmentation before network training. Then, the images are fed into the segmentation networks for training. Finally, we evaluate the performance of the networks on the testing set and visualize the prediction results.

### 3.1. Dataset

In this paper, a large-scale burn dataset was created. We worked with The People's Hospital of Jianggan District, Hangzhou and got 516 unprocessed burn wound images. These images were taken by using cameras and smartphones. The burn images used in this study have been approved by the patients. The privacy parts of the images have also been processed through blurring. The average width of the original images is 3130 pixels, and the average height is 2531 pixels. Because the original size of the images is large, and some of the images contain different burn parts of the patients, we cut the original burn images to expand the burn dataset. And the total number of burn images in the burn dataset was expanded to 1200. Then, the experienced clinical doctors from the hospital labelled the burn areas and the burn depths of the burn images by using LabelMe software developed by Wada [17]. For burn wounds, 5 types were labelled: superficial (S), superficial partial thickness (ST), deep partial thickness (DT), full thickness (FT), and undebrided burn (U). The rest of burn images were classified as the background (B). Considering that most of the burn images collected from the hospital are from patients with severe burns, the labelled areas of superficial and superficial partial thickness are merged into superficial partial thickness. Finally, we got 1200 labelled images of burn wounds. Among them, 960 images are used for training the model and 240 images for testing.  Figure 2 shows part of the burn dataset.  Figure 3 shows an image labelled with LabelMe, and the different colored polygons represent different burn depths. The details of burn depth images and pixels in the training set and testing set are shown in Table 1. The size of each image is resized to 320 × 320 pixels. It can be seen that background pixels occupy the majority, followed by undebrided pixels and deep partial thickness pixels.

### 3.2. Data Augmentation

In the process of model training, we used data augmentation to expand the burn images. Firstly, we flipped the burn images, including horizontal and vertical flips. After that, bilateral filtering, Gaussian blur, and sharpening were used for burn images. Finally, the pseudolabel method [18] was also used for data augmentation. In order to use the pseudolabel method, we first trained a model without data augmentation and then used it to predict the training set. After that, the prediction results (pseudolabels and the pseudolabels of the model were float numbers) and the labels marked by the doctors were averaged as the labels of burn images during training. In this paper, we have designed a total of 6 data augmentation methods for training networks. In the model training process, we used a random number generator to randomly choose whether to use or not to use each data augmentation method for each batch of burn images.

### 3.3. Network Architecture

The network architectures are similar to FCN. The network consists of two main parts: the encoder network and the decoder network. Different backbone networks are selected for the encoder and decoder, including the high-resolution network (HRNetV2) with C1 (one convolution module), residual network-50-dilated (ResNet-50-dilated) with pyramid pooling module (PPM), residual network-101-dilated (ResNet-101-dilated) with pyramid pooling module, residual network-50 (ResNet-50) with unified perceptual parsing network (UPerNet), and residual network-101 (ResNet-101) with unified perceptual parsing network. The encoder networks perform downsampling through convolution to extract semantic feature maps with different resolutions. The decoder networks fuse semantic information of different resolutions through the upsampling operation. And the last layer of the original backbone network (ResNet-50 and ResNet-101) as the encoder is removed. In this paper, bilinear upsampling is used for simplicity.

Figure 4 shows the segmentation network composed of HRNetV2 and C1. HRNetV2 is proposed by Sun et al. [19], and they demonstrate the effectiveness of strong high-resolution representations and multilevel representations learned by the modified networks on semantic segmentation, facial landmark detection, and object detection. We choose HRNetV2 as the decoding network and then connect C1 as the decoding network. The structure of C1 network consists of a convolution layer (kernel size is 3, stride is 1, and padding is 1) and a batch normalization layer with ReLU activation function. From Figure 4, it can be seen that the feature maps of different resolutions are merged at each stage of the HRNetV2 network. Then, the HRNetV2 network outputs 4 feature maps of different sizes in the fourth stage. These feature maps are connected after upsampling and sent to the C1 network. Finally, the output prediction of the C1 network is upsampled to the size of the input image.

Residual networks are presented by He et al. [20]. Through the residual module, they built a series of residual networks. In this paper, we choose ResNet-50 and ResNet-101 as the encoder networks. At the same time, we introduce dilated convolution [21] into ResNet-50 and ResNet-101. The difference between a standard convolution kernel and a dilated convolution is shown in Figure 5. The dilated convolution kernel can get a larger field of view and aggregate multiscale contextual information without loss of resolution. In the original ResNet-50/ResNet-101, the convolution layers (27, 30,…, 42/27, 30,…, 93) are replaced by dilated convolution layers with 2 dilation and the convolution layers (45, 48/96, and 99) are replaced by dilated convolution layers with 4 dilation.

Figure 6 shows the segmentation network composed of ResNet-50-dilated/ResNet-101-dilated and PPM. Pyramid pooling module is a part of the pyramid scene parsing network (PSPNet) which is proposed by Zhao et al. [22] for global scene prior construction upon the final-layer-feature-map of the deep neural network. In this paper, PPM is connected with ResNet-50-dilated/ResNet-101-dilated as the decoding network. PPM performs pooling and convolution operations on the output feature map of the last layer of the ResNet-50-dilated/ResNet-101-dilated network (the last fully connected layer of the original network is removed) at different scales. Then, these feature maps are upsampled and connected to the last layer's feature map of the encoder network. Finally, we perform convolution and upsampling operations on this feature map to obtain the final prediction results.

In the end, we choose the ResNet-50/ResNet-101 as the encoding network and the UPerNet as the decoding network. The unified perceptual parsing network is designed by Xiao et al. [23], which is based on the feature pyramid network (FPN) [24] and pyramid pooling module. FPN uses a top-down architecture with lateral connections to fuse high-level semantic information into middle and low levels. They apply a pyramid pooling module on the last layer of the backbone network before feeding it into the top-down branch in FPN. So, the encoding network does not need dilated convolution which is time and memory consuming [25]. From Figure 7, the four feature maps of ResNet-50-dilated/ResNet-101-dilated are horizontally connected to FPN, and the top feature map is connected to PPM. Finally, the feature maps of different resolutions are connected after upsampling.

### 3.4. Loss Function

In this paper, cross-entropy (CE) loss and focal loss (FL) are used for the training networks. Focal loss was proposed by Lin et al. [26], which applies a modulating term to the cross-entropy loss in order to focus learning on hard negative examples in one-stage object detectors. The cross entropy (CE) loss is

(1) $$\begin{array}{c} \text{CE}\left(y_{\text{pred}},y_{\text{true}}\right)=-\underset{\text{classes}}{\sum }y_{\text{true}}\log\left(y_{\text{pred}}\right). \end{array}$$

In the above, *y*_true_ ∈ {±1} denotes the ground truth class, *y*_pred_ ∈ [0, 1] denotes the network's estimated probability for the class. The focal loss is

(2) $$\begin{array}{c} \text{FL}\left(y_{\text{pred}},y_{\text{true}}\right)=-\alpha {\left(1-y_{\text{pred}}\right)}^{\gamma }\underset{\text{classes}}{\sum }y_{\text{true}}\log\left(y_{\text{pred}}\right), \end{array}$$

where *α* ∈ [0, 1] denotes a factor, which balances the importance of positive and negative examples. *γ* ∈ [0, 5] is also a modulating factor. *α* = 0.25 and *γ* = 2 are chosen in this paper. For superficial partial-thickness, deep partial-thickness, full-thickness, and undebrided burn, the number of pixels of each burn depth category is unbalanced. Therefore, we use the method of median frequency (MF) balancing [27] to weight each burn depth (including the pixels of the background area, because the number of background pixels occupies the majority of the burn dataset). The calculation formula of MF is

(3) $$\begin{array}{c} {\text{MF}}_{c}=\frac{\text{median}\_\text{freq}}{{\text{freq}}_{c}}, \end{array}$$

where freq_*c*_ denotes the number of pixels of class *c* divided by the total number of pixels in images where *c* is present and median_freq denotes the median of these frequencies. Finally, the weighted CE loss and FL are added as total loss (TL):

(4) $$\begin{array}{c} \text{Tota}{\text{l}}_{\text{loss}\left(y_{\text{pred}},y_{\text{true}}\right)}=-\underset{\text{classes}}{\sum }{\text{MF}}_{c}y_{\text{true}}\log\left(y_{\text{pred}}\right)-\alpha {\left(1-y_{\text{pred}}\right)}^{\gamma }\underset{\text{classes}}{\sum }{\text{MF}}_{c}y_{\text{true}}\log\left(y_{\text{pred}}\right). \end{array}$$

### 3.5. Metrics

We use three main metrics to evaluate performance of networks: pixel accuracy (PA), intersection-over-union (IOU), and Dice coefficient (DC). PA measures the proportion of pixels with correct categories to all pixels. IOU, also known as the Jaccard similarity coefficient, measures the ratio of intersection and union between the ground truth area and predicted area of networks. We use mean IOU to evaluate networks for multiple burn depth. Mean IOU is the average of the IOU of each category, which measures the overall performance of networks. DC, or F1 score, measures the similarity between the ground truth and the network's estimated probability. The formulas of three metrics are as follows:

(5) $$\begin{array}{c} \text{Mean PA}=\frac{1}{n}\overset{n}{\underset{i=1}{\sum }}\frac{p_{ii}}{p_{i}},\\ \text{Mean IOU}=\frac{1}{n}\overset{n}{\underset{i=1}{\sum }}\frac{p_{ii}}{p_{i}+\sum_{j=1}^{n}p_{ji}-p_{ii}},\\ \text{DC}=\frac{2\text{TP}}{\text{FP}+2\text{TP}+\text{FN}}, \end{array}$$

where *n* is the number of all classes excluding the background class, *p*_*i*_ is the total number of pixels for class *i*, *p*_*ii*_ is the number of pixels correctly classified for class *i*, and *p*_*ji*_ is the number of pixels of class *i* classified as class *j*. TP is the true positive, which represents the correct pixels of each class. FP is the false positive, which represents the incorrectly pixels of each class. FN is the false negative, which represents the pixels of other classes classified into the class.

## 4. Results

### 4.1. Experiment Setup

Our experiments are carried out on a computer with a NVIDIA GEFORCE RTX-2080Ti GPU with 11 GB memory. The Pytorch deep learning framework is used for training different networks. Part of the training code refers to [28]. The stochastic gradient descent (SGD) is chosen as the optimizer during training, and the initial learning rate of both the encoder and decoder is 0.02. The weight decay is 0.0001, and the learning rate the learning rate will be reduced after each epoch. Before network training, the size of each image is resized to 320 × 320 pixels. The batch size is 8 for training HRNetV2-C1 and ResNet-50-UPerNet. The batch size is 4 for training ResNet-101-UPerNet and ResNet-50-dilated-PPM. And the batch size only is 2 for training ResNet-101-dilated-PPM. Each network is trained for 100 epochs. The initial weights of each network use the pretraining weights on the ImageNet dataset to shorten the training time. For the decoder backbone networks, we remove the last full connection layer of the original networks. For the encoder networks, the size of the output segmentation map is the size of the input size 320 × 320 pixels, and each pixel has multiple channels. The number of the channels is the total number of classes including the background class. The Softmax activation function then is used for each output pixel. During network training, the loss calculation of the output segmentation map and label is performed. In network prediction, the class corresponding to the max value of each pixel channels in the segmentation map will be taken as the predicted class.

### 4.2. Burn or No Burn

We firstly evaluate the performance of the networks in segmenting burn or no burn areas. ST, DT, FT, and U are merged into the burn area. The reason for this is that when labelling the images, the overall burn area is labelled first and then different burn depths are subdivided in this area. The no burn area includes the patient's normal skin pixels and background pixels (the patient's clothes and other pixels are also included). First of all, we want to verify the impact of different loss functions on the network performance. Therefore, we trained the HRNetV2-C1 network with different losses to filter the better loss function. At this stage, no data augmentation strategy is used. The results of the networks on the testing set are shown in Table 2. From Table 2, it can be seen that the performance of the HRNetV2-C1 network with FL is poor. This may be that the attenuation of FL is faster. When the network has not reached the optimum during training, the FL has been reduced to a trivial value that is difficult to optimize. The performance of CE is slightly worse than TL from Table 2. Because TL performs best, we use TL to train the different backbone networks in the subsequent training process.

Table 3 shows the performance of different backbone networks with or without data augmentation. It can be seen that the performance of different backbone networks with data augmentation are better than that without data augmentation. Specifically, the network that performs best on IOU and DC metrics is HRNetV2-C1 with data augmentation. The performance of ResNet-50-dilated-PPM and ResNet-50-UPerNet with data augmentation is slightly inferior to HRNetV2-C1. But ResNet-101-UPerNet without data augmentation achieved the best results on the PA metric, which shows that the network may overpredict the pixels of the burn area. So, we observed the confusion matrix of the two networks ResNet-101-UPerNet no-Aug and HRNetV2-C1 Aug (Tables 4 and 5). It can be seen that ResNet-101-UPerNet no-Aug does over predict the pixels of the burn area. And HRNetV2-C1 is more balanced. Therefore, HRNetV2-C1 is used as the backbone network in the subsequent experiments of multiple burn depths.

After that, we visualize the prediction results of the HRNetV2-C1 Aug network on a part of the testing set, as shown in Figure 8. First of all, the predicted burn area of our network will slightly deviate from the labelled burn area (1, 2, and 3 in Figure 8). In this case, the edges of the burn area are obvious on the whole, but when the burn experts use tools to accurately label, they will find that the edge of the burn area will have a transition from the burned skin to the normal skin. This will produce some human error. And we may not get a very precise label on the edge of the burn area. Secondly, the network will overpredict the burn areas (4, 5, and 6 in Figure 8). Some of the overpredicted areas actually are the burn areas which are not labelled. Some areas are less obvious burn areas with slight redness and some areas with no obvious burn edges. Considering that labelling the burn images may cost a lot of time, it is unlikely that the experts will label all the burn areas. On the other hand, for some burn areas whose edges are difficult to define, burn experts can only subjectively label these areas which are not accurate enough.

### 4.3. Multiple Burn Depth

The best performing network HRNetV2-C1 which is in the previous section is chosen as the backbone network to train a multiburn depth segmentation network. From the burn depth class statistics of the burn dataset (see Table 1), it can be seen that the number of pixels for each burn depth is unbalanced. Therefore, the median frequency-weighted loss function trick is adopted to balance the burn classes. And another initial weight trick is used to train the networks. Specifically, we first train a basic network that does not use data augmentation and weighted loss. Then, the data augmentation and weighted loss is used to retrain the basic network that retains the weights of the first training. The performance of the networks in multiburn depth segmentation is shown in Table 6. It can be seen that when using the data augmentation strategy to train the network, the performance of the network on the metrics of mean IOU, mean PA, and mean DC is better than the basic network without data augmentation. When the weighted loss function is used or the weight of the basic network is used to retrain a new network, the performance of networks does not improve significantly. Although the network trained by using data augmentation and basic model weight achieves the best performance in different metrics, it cannot widen the gap between the models trained with other strategies.  Figure 9(a)–9(c) show the performance of the networks on IOU, PA, and DC in each burn depth class. The performance of the networks with different strategies in each burn depth class is not much different. Although we want to improve the imbalance of different burn depth classes by using a weighted loss strategy, the results of experiment show that the effect of this strategy is not obvious. And when using the strategy of the basic model weight to retrain a network, the new network does not perform better than others in testing set.

Table 7 shows the confusion matrix of the Aug & Basic_Weight network on testing set pixels. From Table 7, we find that the incorrectly predicted pixels of superficial partial thickness burns are mainly classified as background, deep partial-thickness burns, and undebrided burns, but there are fewer pixels that are incorrectly classified as full-thickness burns. The incorrectly predicted pixels of deep partial thickness are mainly classified as undebrided burns. And the incorrectly predicted pixels of full-thickness burns are mainly classified as deep partial thickness. As a result, the network is better at distinguishing superficial partial thickness from full thickness and superficial partial thickness from undebrided burns, which may be the characteristics of these classes with obvious differences. However, the network poorly distinguishes superficial partial thickness from deep partial thickness, deep partial thickness from full thickness, and deep partial thickness from undebrided burn, which may be because the characteristics between them are similar.

Figure 10 shows the visual prediction results of the HRNetV2-C1 network (Aug & Basic_Weight) on a part of the testing set. First, the network performs better in segmenting burn areas, but the prediction of burn depth in some areas is sometimes wrong (1 in Figure 10). Secondly, for burn areas with complex depths (2–6 in Figure 10), the boundaries between different burn depths are not clear, which more is the transition from superficial burns to deep burns. In this case, burn experts are more inclined to label entire burn area and then diagnose the depth of the burn area as a whole. However, the network will segment other burn depth areas in the entire burn area. Therefore, this data annotation problem will have a negative impact on the network performance. In fact, burn experts are unlikely to have enough energy to label all burn areas in detail and diagnose the burn depth. So, the entire training process needs to be shifted to a semisupervised process. We can assume that the data annotation is incomplete. After first training the networks, the segmentation results of the networks can be fed back to the burn expert. Then, the burn expert can decide whether the prediction results of the network can be used as a new segmentation label. Finally, the new labelled dataset is used to train the model to form a feedback loop.

## 5. Discussion

The foundation of automatic burn diagnosis is the segmentation of the burn image area. Accurate segmentation of the burn area and prediction of burn depth provide important help for the following clinical treatment. In this paper, we propose an end-to-end advanced burn area segmentation and burn depth diagnosis framework. First of all, our network has achieved satisfactory results in segmenting the burn or no burn areas. Furthermore, this network framework for segmenting burn areas can be easily extended to a network for segmenting normal skin and burned skin areas. If we label the normal skin area in the burn dataset for network training, the network will segment both the normal skin and the burn skin. And, if a whole body burn image is taken from a patient, we can calculate the percentage of the burn area in TBSA through this network and then diagnose the severity of burn.

After that, we evaluate the performance of the network on multiple burn depth segmentation. However, in the end-to-end multiple burn depth segmentation, the performance of the network did not surprise us. Although some strategies can improve the performance of the network, the improvement is limited. When we observe the confusion matrix predicted by the network, we find that the prediction results are poor for areas with similar burn depths (such as deep partial thickness and full thickness). Because of the imbalance in the number of pixels of different burn depths, most of the incorrect pixels predicted by the network are background and undebrided burns. By visualizing the prediction results of the network, we find that the semisupervised learning paradigm may improve the labelling of the burn dataset and the training process of the network. When the labelling of the burn dataset is more accurate, the performance of the network may be further improved.

## 6. Conclusions

In this paper, an end-to-end framework for burn area segmentation and burn depth diagnosis based on deep learning is proposed. First, we build a large-scale burn dataset with detailed segmentation and annotation. After that, data augmentation and other strategies are used to improve the performance of the network models. Then, the total loss function is used to train the network models. Finally, the IOU, PA, and DC metrics are used to evaluate the performance of the network models. And the prediction results of the network models are visualized. In the segmentation for the burn and no burn areas, the networks have a good performance and, respectively, achieve the best results of 0.8467, 0.9459, and 0.9170 on the IOU, PA, and DC metrics. And only by simply expanding the network structure and labelling the burn dataset, we may easily train a network of segmenting burn skin and normal skin to calculate the percentage of burns in TBSA, which has a high clinical value. After that, the networks obtain a mean IOU of 0.5144, a mean PA of 0.6684, and a mean DC of 0.6782 in the multiple burn depth segmentation. In total, this burn diagnosis framework will provide important help for clinical burn diagnosis and treatment.

## Figures and Tables

**Figure 1:** The deep learning burn diagnosis framework.

**Figure 2:** Examples of burn images in the burn dataset.

**Figure 3:** A burn image annotated with LabelMe.

**Figure 4:** HRNetV2 and C1 networks. (b–e) The 1st, 2nd, 3rd, and 4th stages of HRNetV2, respectively,. The upward arrow refers to the upsampling process, the horizontal arrow refers to the size of feature maps remaining unchanged after convolution, and the downward arrow refers to the downsampling convolution.

**Figure 5:** Dilated convolution with 3 × 3 kernel size and different dilation rates. The standard convolution kernel can be regarded as a dilated convolution with dilation rate of 1. The expansion rate from (a) to (c) is 1, 2, and 4.

**Figure 6:** The network structure composed of ResNet-50-dilated/ResNet-101-dilated and PPM.

**Figure 7:** The segmentation network composed of ResNet-50/ResNet-101 and UPerNet. The four feature maps of ResNet-50/ResNet-101 on the left feature pyramid are the output of the 10th, 22nd, 40th and 49th/10th, 22nd, 91st, and 100th convolutional layers. The sizes of the four downsampling feature maps, respectively, are 1/4, 1/8, 1/16, and 1/32 of the original input image size.

**Figure 8:** Examples of burn areas predicted by the network. Blue indicates burn areas, and black indicates no burn areas.

**Figure 9:** The performance of the networks on IOU, PA, and DC in different burn depth classes.

**Figure 10:** Examples of the network segmentation of multiple burn depth areas. Blue indicates superficial partial-thickness burn, green indicates deep partial-thickness burn, red indicates full-thickness burn, yellow indicates undebrided burn, and black indicates background area.

**Table 1:** The number of pixels and images corresponding to each burn depth category in the burn dataset. Because each image may contain different burn depths, the total number of images in the table is larger than the number of images in the burn dataset.

	B	ST	DT	FT	U
Training set pixels	46,074,508	5,810,773	15,340,840	9,384,514	21,693,365
Training set images	947	168	685	374	510
Testing set pixels	12,906,802	1,874,803	2,908,626	2,758,834	4,126,935
Testing set images	239	44	100	82	97

**Table 2:** Results of HRNetV2-C1 networks trained with different loss on testing set.

Loss	IOU	PA	DC
CE	0.8288	0.9301	0.9064
FL	0.7905	0.9000	0.8830
TL	0.8308	0.9331	0.9076

**Table 3:** Results of different backbone networks on testing set.

	IOU	PA	DC
HRNetV2-C1 no-Aug	0.8308	0.9331	0.9076
HRNetV2-C1 Aug	0.8467	0.9403	0.9170
ResNet-50-dilated-PPM no-Aug	0.8136	0.9231	0.8972
ResNet-50-dilated-PPM Aug	0.8412	0.9374	0.9138
ResNet-50-UPerNet no-Aug	0.8147	0.9321	0.8979
ResNet-50-UPerNet Aug	0.8341	0.9375	0.9096
ResNet-101-dilated-PPM no-Aug	0.7864	0.9215	0.8804
ResNet-101-dilated-PPM Aug	0.7913	0.9128	0.8835
ResNet-101-UPerNet no-Aug	0.8162	0.9459	0.8988
ResNet-101-UPerNet Aug	0.8259	0.9172	0.9046

**Table 4:** The confusion matrix of ResNet-101-UPerNet no-Aug on the testing set pixels.

		Predicted	
		No burn	Burn
Actual	No burn	10,919,332	1,872,931
	Burn	637,499	11,146,238

**Table 5:** The confusion matrix of HRNetV2-C1 Aug on the testing set pixels.

		Predicted	
		No burn	Burn
Actual	No burn	11,490,505	1,301,758
	Burn	703,644	11,080,093

**Table 6:** The performance of the HRNetV2-C1 networks trained with different training strategies on the testing set. HRNetV2-C1 Base means that no training strategy is used. HRNetV2-C1 Aug means that data augmentation is used. Aug & Weighted_Loss means that data augmentation and weighted loss strategies are used. Aug & Basic_Weight means that data augmentation and basic model weight strategies are used. The background class is not included when calculating mean IOU, mean PA, and mean DC.

	Mean IOU	Mean PA	Mean DC
HRNetV2-C1 Base	0.4732	0.6389	0.6413
HRNetV2-C1 Aug	0.5118	0.6578	0.6757
Aug & Weighted_Loss	0.5106	0.6615	0.6739
Aug & Basic_Weight	0.5144	0.6684	0.6782

**Table 7:** The confusion matrix of the Aug & Basic_Weight network on the testing set pixels.

		Predicted				
		B	ST	DT	FT	U
Actual	B	11,765,286	188,437	188,241	76,533	688,305
	ST	245,702	1,118,455	261,268	7,470	241,908
	DT	169,071	101,038	1,924,161	252,898	461,458
	FT	188,077	49,451	613,401	1,717,410	190,495
	U	442,907	73,143	253,889	84,268	3,272,728

## Data Availability

The data during the current study are available from the corresponding author on reasonable request.
